# Effect of Blood Homocysteine on the Outcome of Artificial Insemination in Women with Polycystic Ovary Syndrome

This article has been retracted.

**DOI:** 10.1155/2022/6311419

**Published:** 2022-08-21

**Authors:** Jing Cao, Haiyan Wang

**Affiliations:** The First Affiliated Hospital of Xi'an Jiaotong University, Xi'an, 710061 Shaanxi, China

## Abstract

**Background:**

Polycystic ovary syndrome (PCOS) is the major reason for women's low fertility and the most frequent endocrine disorder in women of childbearing age. Homocysteine is an amino acid that contains sulfur that has been negatively correlated with the reproductive outcome of polycystic women treated with IVF/ICSI. However, the impact of blood homocysteine levels on the outcome of artificial insemination in polycystic ovary syndrome women is unknown. The goal of this study is to examine the impact of serum homocysteine on the result of intrauterine insemination in females who have polycystic ovary syndrome (PCOS).

**Methods:**

96 infertile women (129 cycles) treated with artificial insemination were collected, including 66 cases (87 cycles) in the case group (PCOS group) and 30 cases (42 cycles) in the control group (male factor infertility). The differences in general data amongst two groups, such as BMI, Hcy, and age, were compared. The case group has been classified into two groups based on serum Hcy level: LHcy group (Hcy < 15) and HHcy group (Hcy ≥ 15). The relationship among pregnancy and serum Hcy level outcome in PCOS women was compared.

**Results:**

The PCOS group had substantially increased serum homocysteine levels in comparison to the control group (*P* = 0.019). Among PCOS women, the clinical pregnancy rates of artificial insemination in the HHcy group and LHcy group were 14.29% and 37.88%. The difference among the two groups was substantial (*P* = 0.044). Artificial insemination frequency, ovulation induction, BMI, infertility years, AMH, serum testosterone, HOME IR, TSH, TPOAb, hCG, daily follicle size, intimal thickness, and other factors did not differ greatly between the two groups.

**Conclusion:**

Serum homocysteine levels are increased in women having PCOS. Their levels above the threshold will lower the clinical pregnancy rate of intrauterine insemination in PCOS women.

## 1. Introduction

Polycystic ovary syndrome (PCOS) is a multisystem and comprehensive disease involving reproduction, cardiovascular disease, endocrine disorder, and metabolism. Polycystic ovary syndrome causes symptoms in nearly 5-10 percent of childbearing age women. It is considered to be one of the main reasons for the low fertility of women. Besides, for women of childbearing age, it is the most frequent endocrine problem [1, 2]. The clinical manifestations include highly heterogeneous, mainly characterized by rare ovulation or anovulation, polycystic ovarian changes, and hyperandrogenemia, accompanied by metabolic disorders, such as insulin resistance and lipid metabolism disorder, increasing the long-term cardiovascular risk [3, 4].

Artificial insemination is an assisted reproductive technology (ART), which is utilized for treating infertility occurred through mild to moderate endometriosis, male factors, unexplained factors, and ovulation failure. It can improve the pregnancy rate of PCOS women who have not been pregnant after repeated ovulation induction. IUI refers to the direct injection of washed sperm into the uterine cavity through the cervix and is one of the commonly used artificial insemination techniques. IUI is a safer, simpler, and less expensive treatment option in comparison to in vitro fertilization (IVF)/intracytoplasmic sperm injection (ICSI) [5, 6].

Homocysteine (Hcy) is an amino acid that contains sulfur and exists in two pathways of remethylation and trans-vulcanization in order to form cysteine and methionine [7, 8]. Folic acid, vitamin B12, and vitamin B6 are required in amino acid metabolism as cofactors in various phases of the pathway [7]. Several researches have indicated that serum homocysteine level in polycystic ovary syndrome women is greater in comparison to that in non-PCOS women [7, 9–12]. The presence of PCOS is accompanied by a 23% increase in Hcy levels [13], which may be related to hyperinsulinemia [14]. High homocysteine levels in PCOS women were linked to abortion, ovulation disturbance, as well as decreased embryo quality during ART [10, 11, 15]. However, there is a paucity of research on the link between the outcome of artificial insemination and a high HCY level in PCOS women. This study intends to explore how HCY levels affect artificial insemination outcomes in PCOS women.

## 2. Materials and Methods

### 2.1. Participants

From January 2020 to December 2021, 96 women (129 cycles) who received intrauterine insemination- (IUI-) assisted pregnancy in the First Affiliated Hospital of Xi'an Jiaotong University were collected, including 66 cases (87 cycles) in the case group (PCOS group) and 30 cases (42 cycles) in the control group (male factor infertility). The patients' general status, serum Hcy level, and sex hormone status of the 2nd-4th day of menstrual period, thyroid stimulating hormone (TSH), Anti Mullerian Hormone (AMH), male semen, thyroid peroxidase antibody (TPOAb), salpingography, and other data; fasting insulin levels and fasting blood glucose were used to determine the degree of insulin resistance, with home IR = fasting blood glucose (mIU/L) × fasting insulin (mmol/L)/22.5. Couples with age ≥ 35 or AMH ≤ 1.1 and bilateral AFC<7, complicated with endometriosis, intrauterine lesions were excluded. Based on the 2003 revised Rotterdam criteria, after eliminating other probable disorders that mirror the polycystic ovary syndrome phenotype, it is diagnosed when two out of three of the conditions given below are present: (1) biochemical and/or clinical symptoms of hyperandrogenism, (2) polycystic ovaries on ultrasound examination, and (3) oligo and/or anovulation [16]. Then, the case group was classified into two groups based on the serum Hcy level, the HHCY group (Hcy ≥ 15), and the LHCY group (Hcy < 15). The relationship among pregnancy outcome and serum Hcy level in PCOS women was compared.

### 2.2. Methods

In the IUI procedure, ovulation was monitored by natural cycle or stimulated by letrozole/HMG. Natural cycle is applicable to women who have ovulation; from the 9th day of menstrual cycle, ovulation is monitored by vaginal B-ultrasound. Ovulation induction is applicable to anovulatory women. Letrozole 2.5-5.0 mg/day is taken orally from the 4th to 5th day of menstrual cycle, and vaginal B-ultrasound is performed after 5 days; if there is no ovarian response, HMG75 IU/day is added; or directly apply HMG75 IU/day from the 4th to 5th day of menstrual cycle. Carry out regular transvaginal ultrasound monitoring of follicular development and adjustment of HMG dosage.

When follicle diameter ≥ 18 mm or the urinary luteinizing hormone test is positive, combine serum LH, E2, and P values for the purpose of determining whether to continue injecting urinary human chorionic gonadotropin (HCG) 6000-10000IU. 24 hours after the trigger, vaginal B-ultrasound was performed so as to monitor ovulation, and the first intrauterine artificial insemination was performed; if ovulation occurred, luteal support was given; if there is no ovulation, B-ultrasound is performed again 24 hours after the operation, and IUI was performed for the second time following ovulation.

After ovulation, all patients have treated with didroxyprogesterone tablets of 20-30 mg/day for supporting the corpus luteum. Prior to ovulation, if the intima is ≤7 mm, give estradiol valerate 1-3 mg/day. Blood/urine HCG was detected 14 days after the operation to assess whether the patient was pregnant. If pregnant, the corpus luteum continued to support to 10 weeks of pregnancy. One month after the operation, vaginal ultrasonography revealed that gestational sac and fetal heartbeat were defined as clinical pregnancy. Follow up 10 weeks after the operation to check if there was an abortion. If not, a B-ultrasound examination was undertaken to confirm whether there was continuous pregnancy.

### 2.3. Statistical Analysis

For data statistics, SPSS25.0 statistical software was used; the measurement data has been first tested by the Shapiro-Wilk test for normality, normal distribution's measurement data were expressed by mean ± standard deviation (*x* ± *s*), and the mean of the two samples was compared using an independent sample test. The quartile and median [*M*(P25, P75)] were used to express measurement data that did not fit into a normal distribution, and the Mann–Whitney *U* test was used to compare the two sample levels. The counting data were represented by sample rate or frequency, and the groups were compared using the chi-square test. *P* < 0.05 pointed out that the difference was statistically substantial.

## 3. Results

### 3.1. Disease Characteristics of PCOS

There were 66 females in the PCOS group and 30 females in the control group; the clinical characteristics, as well as the general data amongst the two groups, are presented in Table 1. Between the two groups, there was no discernible age difference. The infertility years in the polycystic ovary syndrome group were longer in comparison to the control group, which may be related to the fact that the PCOS group received more excretion-promoting therapy and was transferred to artificial insemination after several cycles of failure to pregnancy. The BMI of the PCOS group was higher in contrast to the control group; however, the difference was not significant. The levels of AMH, AFC, and serum T in the polycystic ovary syndrome group were more in contrast to the control group (*P* < 0.05), which was consistent with the disease characteristics of PCOS; vitamin B12 and serum levels were not significantly different among two groups; however, the level of serum Hcy in PCOS group was substantially higher in contrast to the control group (*P* = 0.019). TSH and TPO-Ab levels did not differ significantly among the two groups. The level of FSH in the control group was slightly higher on the 2nd-4th day of menstrual period, and there was no significant difference in E2 and LH levels (Table 1).

### 3.2. Analysis of the General Situation of Women with Hcy-Stratified PCOS and the Pregnancy Outcome of Husband Sperm Artificial Insemination

According to the level of serum Hcy, they were classified into two groups: the HHcy group (Hcy ≥ 15) and the LHcy group (Hcy < 15). The LHcy group was slightly older than the HHcy group in terms of age. BMI, years of infertility, AMH, E2, FSH, LH, home IR, TSH, TPOAb, HCG daily follicular size, and intimal thickness were not significantly different between the two groups. The HHcy group had lower VitB12 and serum folate levels than the LHcy group, with no substantial difference among the two groups. The overall number of husband's forward motile sperm did not differ between the two groups (see Table 2).

Between the two groups, there was no difference in ovulation mode and IUI frequency. The clinical pregnancy rate in the LHcy group (37.88%) was significantly higher than that in the HHcy group (14.29%). There was a significant difference among the two groups (*P* < 0.05). The abortion rate in the HHcy group (33.33%) was higher in comparison to the LHcy group (12%), although there was no statistically significant difference between the two groups (see Table 3).

## 4. Discussion

PCOS is a multisystem, comprehensive, and complex disorder that affects reproduction, the endocrine system, cardiovascular system, and metabolism. It is one of the main reasons for low fertility as well as the most frequent endocrine problem in childbearing age women [1, 2]. At present, the etiology of PCOS is unclear; however, genetic and environmental factors may play a role [11]. The clinical manifestations of polycystic ovary syndrome are highly heterogeneous, mainly characterized by rare ovulation or anovulation, polycystic ovarian changes, and hyperandrogenemia, combined with metabolic problems such as insulin resistance, seriously affecting the fertility of patients and increasing the long-term cardiovascular risk [3, 4].

Homocysteine is an amino acid that contains sulfur and is an intermediate product of methionine metabolism. After the methionine in food enters the human body, it generates S-adenosylmethionine under the catalysis of methionine adenosyltransferase. After S-adenosylmethionine is methylated, it can form S-adenosylhomocysteine, which releases adenosine after hydrolysis in order to generate Hcy [8]. Hcy is primarily metabolized through remethylation and trans-vulcanization; besides, a small amount of Hcy is synthesized in cells and directly released into plasma [8]. Increased serum homocysteine can be caused by genetic defects of enzymes implicated in the homocysteine pathway, for instance, methylenetetrahydrofolate reductase (MTHFR), deficiency of vitamin cofactors like vitamin B12, folic acid, and vitamin B6 or the influence of drugs such as Bates and niacin [17–20]. Hyperhomocysteinemia (HHcy) is generally regarded as an independent risk factor for atherosclerosis and thromboembolism, whereas PCOS also has a long-term risk of cardiovascular disease [7, 8]. As revealed by the previous literatures, the level of homocysteine is considerably enhanced in polycystic ovary syndrome (PCOS) patients [[7, 9–12]]. In addition to the possible correlation between Hcy level and metabolic syndrome, there are a variety of interfering factors, such as vitamin B12, folic acid, vitamin B6 levels, and genetic enzyme deficiency [17–20]. In this study, in contrast to the control group, patients having PCOS had increased levels of Hcy when vitamin B12, BMI, and serum folate levels were balanced. This also supports the presence of an association among PCOS and Hcy patients, and high Hcy levels may be a disease feature of PCOS.

Insulin resistance refers to the phenomenon caused by a variety of reasons insulin in the body which reduces the efficiency of promoting glucose into the tissue, raises blood glucose, and leads to the compensatory increase of insulin in the body. It can be found in up to 70% of PCOS women [12]. It is one of the important characteristics of PCOS, and it participates in the PCOS pathological procedure [12]. Pat research has indicated that the increase of Hcy level in PCOS women has nothing to do with obesity and hyperandrogen, but is related to insulin resistance [11, 13, 14, 21]. In patients having polycystic ovary syndrome, the number of CD14CD16 inflammatory monocytes in peripheral blood with hyperhomocysteinemia increases. CD14CD16 monocytes may play a role in the pathogenesis of insulin resistance in PCOS patients [22]. High insulin levels can be achieved through inhibition of hepatic cystine *β* or glomerular filtration [11]. However, IR, age, and BMI according to some studies are not associated with the level of Hcy in PCOS women [23]. Metformin treatment did not lower Hcy levels in PCOS patients, especially in women with BMI > 25 kg/m^2^ [24]. In this study, no significant disparity was found in BMI, home IR, and blood testosterone between LHcy and HHcy groups, and even BMI and home IR in the LHcy group were somewhat higher in comparison to in the HHcy group. However, the HHcy group had relatively lower vitamin B12 and folic acid levels. This suggests that Hcy, as a member of Vit B12 and folate metabolic pathway, might be a risk factor independent of IR, androgen level, and BMI in PCOS women. It can be further studied after expanding the sample and balancing the influencing factors such as vitamin B12 and folic acid levels.

Previous research has revealed that artificial insemination's pregnancy outcome is related to age, endometrial thickness, ovulation induction, the total number of forward sperm, frequency of artificial insemination, and so on [6]. According to prior research, homocysteine level in follicular fluid is negatively correlated with pregnancy outcome as well as embryo quality in patients receiving IVF/ICSI [15, 25]. High levels of Hcy have direct cytotoxicity, which may cause intimal damage, excessive production of oxidative stress substances (ROS), inhibition of methylation, and abnormal gene expression [15, 26, 27]. High levels of Hcy could result in follicular occlusion, thus reducing oocytes' quality, number, and developmental potential, impacting the quality of embryo implantation, early embryos, and pregnancy maintenance [10, 15]. Hcy will produce free radicals and hydrogen peroxide, along with other products in the oxidation process, which will not only damage vascular endothelial cells, but likewise inhibit the synthesis and release of nitric oxide in vascular endothelial cells, increase the damaging effect of lipid peroxide on cells, and eventually interfere with and destroy the integrity of endometrial blood vessels [15]. Other influencing factors related to the pregnancy rate of artificial insemination, such as ovulation induction, endometrial thickness, artificial insemination frequency, and the total number of forward motile sperm of the husband, were not different between the two groups, and even though the age of LHcy group was slightly greater in contrast to HHcy group, which is not conducive to pregnancy. But the clinical pregnancy rate in the LHcy group (37.88%) and HHcy group (14.29%), there was a considerable difference among the two groups (*P* < 0.05). Therefore, the level of homocysteine exceeding the threshold could significantly reduce the pregnancy rate of artificial insemination in PCOS women.

The abortion rate induced by hyperhomocysteinemia, based on prior research is significantly greater than the normal blood group cysteine segment [30, 31]. Hcy can inhibit the expression of thrombomodulin, interfere with protein C regulation related to endothelial cells, decrease the activity of antithrombotic factor VI and factor VII, increase the activation of thrombin by coagulation factors V and Xa, destroy the balance between fibrinolysis and coagulation, and make the body in a prethrombotic state; Hcy can likewise cause direct thrombosis and endothelial injury via oxidative stress response [14, 23]. Under the action of the above two mechanisms, the risk of villous thrombosis increases, and the risk of spontaneous abortion also increases [28–30]. In this study, although the abortion rate in the HHcy group is not statistically different from that in the LHcy group, the abortion rate in the HHcy group (33.33%) is higher in comparison to that in the LHcy group (12%), which may be due to the small amount of data and the usage of aspirin in a patient with the hypercoagulable state during pregnancy, so Hcy levels above the threshold may be detrimental to the maintenance of pregnancy.

In summary, patients with PCOS had increased homocysteine levels in comparison to the control group. The high Hcy level in PCOS women was related to vitamin B12 and serum folate levels, however, not to insulin resistance, Kaohsiung, and BMI; hyperhomocysteinemia can reduce the pregnancy rate of artificial insemination in PCOS patients. Therefore, this paper believes that Hcy is an independent factor affecting the outcome of PCOS artificial insemination. In order to predict the outcome of PCOS in female artificial insemination, we should improve the understanding of Hcy, actively detect, early treat, and intervene in clinical work, so as to improve the pregnancy rate and reduce early pregnancy loss.

## Figures and Tables

**Table 1:** Disease characteristics of PCOS.

	PCOS group (*n* = 66)	Control group (*n* = 30)	*Z*/*t*	*P*
Age (years)	29.39 ± 3.16	30.6 ± 2.84	-1.787	0.077
Years of infertility	2 (1, 4)	1 (1, 3)	-2.044	0.041
BMI	23.69 ± 3.67	22.28 ± 3.29	1.803	0.075
AMH	6.48 (4.63, 7.18)	2.84 (1.99, 3.72)	-6.817	<0.001
AFC	24 (23, 24)	15 (10, 19)	-7.442	<0.001
E2	121.00 (102.85, 175.78)	117.60 (106.85, 160.80)	-0.158	0.874
T	1.04 (0.71, 1.35)	0.79 (0.48, 1.08)	-2.720	0.007
FSH	6.22 (5.27, 7.09)	7.15 (6.08, 7.64)	-2.316	0.021
LH	5.36 (4.04, 7.61)	5.39 (4.21, 6.8)	-0.316	0.752
HCY	12.10 (9.78, 14.70)	10.45 (8.95, 11.55)	-2.352	0.019
Folate	13.68 (7.86, 19.76)	15.64 (9.86, 20)	-0.676	0.499
Vitb12	373.90 (290.23, 498.93)	444.70 (347.15, 608.83)	-1.684	0.092
TPOAb	13.98 (9.18, 22.37)	12.13 (8.11, 22.29)	-0.957	0.339
TSH	2.51 (1.67, 3.38)	2.28 (1.61, 2.73)	-1.051	

**Table 2:** The general situation of women with Hcy-stratified polycystic ovary syndrome.

	LHcy (*n* = 50)	HHcy (*n* = 16)	*Z*/*t*	*P*
Age (years)	29.9 ± 3.15	27.81 ± 2.71	2.380	0.020
Years of infertility	2 (1, 3)	2 (1.5, 5)	-0.414	0.679
BMI	23.86 ± 3.62	23.16 ± 3.90	0.661	0.511
Home-IR	2.77 (1.91, 5.53)	2.30 (1.50, 4.61)	-1.257	0.209
AMH	6.54 (4.58, 7.29)	5.91 (5.22, 7.14)	-0.914	0.361
AFC	23.54 ± 2.37	22.63 ± 2.13	1.378	0.173
E2	135.55 (104.05, 182.5)	115.05 (84.45, 143.40)	-1.609	0.108
T	1.04 (0.64, 1.40)	1.03 (0.76, 1.31)	-0.247	0.805
FSH	6.17 (5.27, 6.93)	6.73 (5.23, 7.49)	-1.152	0.249
LH	5.44 (4.20, 8.17)	4.82 (3.76, 7.08)	-0.875	0.381
Follicle size	19.05 ± 1.84	18.78 ± 1.18	0.546	0.587
Intimal thickness	9.23 ± 1.99	10.00 ± 2.03	-1.339	0.185
HCY	10.90 (9.25, 12.23)	20.05 (16.70, 29.45)	-5.987	<0.001
Folate	15.57 (11.01, 20.00)	7.45 (5.79, 15.27)	-3.353	0.001
Vitb12	415.70 (316.83, 551.70)	276.20 (241.28, 351.28)	-3.801	<0.001
TPOAb	15.00 (9.53, 23.08)	12.90 (7.59, 16.43)	-0.950	0.342
TSH	2.50 (1.59, 3.28)	2.68 (1.70, 3.94)	-0.688	0.491
Forward motile sperm of husband	97.77 (56.82, 155.00)	101.98 (50.81, 171.08)	-0.209	0.834

**Table 3:** Homocysteine stratified PCOS female artificial insemination outcome.

	LHcy (*n* = 66)	HHcy (*n* = 21)	*Z*/*χ*^2^	*P*
Ovulation (*n*/%)			2.354	0.149
No	3 (4.55)	3 (14.29)		
Yes	63 (95.45)	18 (85.71)		
Times of IUI (*n*/%)			-1.059	0.290
1	9 (13.63)	5 (23.81)		
2	57 (86.36)	16 (76.19)		
Pregnancy outcome (*n*/%)			4.063	0.044
Not clinical pregnancy	41 (62.12)	18 (85.71)		
Clinical pregnancy	25 (37.88)	3 (14.29)		
	LHCY group pregnancy (*n* = 25)	HHCY group pregnancy (*n* = 3)	*χ* ^2^	*P*
Abortion (*n*/%)	3 (12)	1 (33.33)	0.996	0.382

## Data Availability

No data were used to support this study.
